# Diagnostic and Prognostic Value of DACH1 Methylation in the Sensitivity of Esophageal Cancer to Radiotherapy

**DOI:** 10.1155/2022/6857685

**Published:** 2022-09-29

**Authors:** Jing Huang, Weiguo Zhu, Wanwei Wang, Yingying Xu, Lei Jiang, Zhenlin Gu

**Affiliations:** ^1^Department of Radiation Oncology, The Affiliated Huaian No.1 People's Hospital of Nanjing Medical University, Huaian 223300, Jiangsu, China; ^2^Department of Vascular Surgery, The Affiliated Huaian No.1 People's Hospital of Nanjing Medical University, Huaian 223300, Jiangsu, China

## Abstract

To detect the methylation status of the cell fate determinant (DACH1) gene in esophageal cancer tissues and to explore the predictive value of methylation of DACH1 on the sensitivity to radiotherapy for esophageal cancer. Cancer tissues, corresponding paracancerous tissues, and 30 specimens of normal esophageal mucosal tissues from 70 patients admitted to the hospital after radical esophageal cancer radiotherapy from January 2016 to April 2017 were collected. The methylation status of DACH1 was detected by a methylation-specific polymerase chain reaction (MSP). The 70 esophageal cancer patients were divided into radiotherapy-sensitive and radiotherapy-insensitive groups according to the efficacy of radiotherapy, and the methylation status of DACH1 was compared between the two groups. The *χ*^2^ test was used to analyze the relationship between the methylation status of DACH1 and the clinicopathological characteristics of esophageal cancer patients. The Kaplan–Meier survival curve was used to analyze the relationship between the methylation status of DACH1 and radiotherapy sensitivity and survival of esophageal cancer patients, and the Cox proportional risk model was used to analyze the independent influencing factors affecting the radiotherapy sensitivity of esophageal cancer patients. The methylation rate of DACH1 in esophageal cancer tissues was higher than that in paracancerous tissues and normal tissues, and the differences were statistically significant (*P* < 0.05). 70 patients with esophageal cancer completed radiotherapy, including 46 patients with radiotherapy sensitivity and 24 patients with radiotherapy insensitivity. The DACH1 methylation rate of esophageal cancer patients in the radiotherapy-sensitive group was lower than that in the radiotherapy-insensitive group, and the difference was statistically significant (*P* < 0.05). The DACH1 methylation rate of esophageal cancer patients with TNM stage (III-IV), tumor differentiation degree (hypofractionation), and lymph node metastasis was higher, and the difference was statistically significant (*P* < 0.05). The Kaplan–Meier curve showed that the median survival time of patients with DACH1 methylation before radiotherapy was 23 months, which was shorter than that of patients with DACH1 unmethylation before radiotherapy (36 months), and the difference between the survival curves of the two groups was statistically significant (*χ*^2^ = 7.425, *P* < 0.05); the median survival time of patients in the radiotherapy-sensitive group was 39 months, which was longer than that of patients in the radiotherapy-insensitive group (25 months), and the difference between the two groups was statistically significant (*P* < 0.05). The median survival time of patients in the radiotherapy-sensitive group was 39 months, which was longer than that of patients in the radiotherapy-insensitive group (25 months), and the difference in survival curves between the two groups was statistically significant (*χ*^2^ = 7.011, *P* < 0.05). The results of the multifactorial Cox regression model showed that TNM stage (stage III-IV) (HR = 1.961, 95% CI: 1.125–2.768), tumor hypofractionation (HR = 1.453, 95% CI: 1.034–2.857), presence of lymph node metastasis (HR = 1.499, 95% CI: 1.025–2.851), and DACH1 methylation (HR = 1.718, 95% CI: 1.067–2.596) may increase the risk of insensitivity to radiotherapy in patients with esophageal cancer (*P* < 0.05). The rate of DACH1 methylation in esophageal cancer tissues was increased, and the methylation status of DACH1 was related to radiotherapy sensitivity and survival of esophageal cancer patients, which is expected to be a new target for diagnosis and treatment of esophageal cancer patients.

## 1. Introduction

Esophageal cancer is one of the most common malignant tumors in clinical practice. In its early stages, it can have the feeling of a foreign body in the pharynx. With the increase of tumor volume and the progress of the disease, it can have typical progressive symptoms such as eating obstruction, pharyngeal sensation, and poststernal pain after eating. The incidence rate of esophageal cancer ranks seventh among the incidence rates of malignant tumors in the world, and it is also the sixth most common cause of cancer death [1]. China is one of the regions with the highest incidence of esophageal cancer in the world, with the fifth highest incidence rate and an average of about 150,000 deaths per year, among which esophageal squamous cell carcinoma accounts for up to 90% of the deaths and is the deadliest type [2]. Most patients with esophageal cancer have no obvious early symptoms and are already in the middle to late stages when they are diagnosed, losing the best opportunity for surgery [3]. The carcinogenesis and development mechanism of esophageal cancer is a complex process involving the accumulation and interaction of multifactor, multistage, and multigene mutations. This process may occur at the level of genomic DNA, mRNA, or protein. In recent years, molecular biology research on the mechanism of esophageal cancer suggests that this process presents a multistage evolution, accompanied by the interaction and superposition of multiple genes, especially the activation of oncogenes and the inactivation of tumor suppressor genes, which is an important basis for abnormal cell proliferation and carcinogenesis. The molecular biological mechanisms of cell cycle regulation, signal transduction, cell differentiation, damage repair, and apoptosis are indispensable factors leading to the occurrence and development of tumors. Therefore, exploring the biological mechanism of esophageal cancer radiotherapy sensitivity and finding novel markers that can predict the sensitivity of esophageal cancer radiotherapy has become a current research hotspot. Molecular mechanism studies have shown that the development of esophageal cancer is closely related to genetic and epigenetic genetic alterations. Epigenetics is a branch of genetics that studies the heritable changes in gene expression without changing the nucleotide sequence of genes. There are many epigenetic phenomena, including DNA methylation, genomic imprinting, maternal effect, gene silencing, nucleolar dominance, dormant transposon activation, and RNA editing. DNA methylation is the most common epigenetic alteration involving the activation of oncogenes and inactivation of oncogenes. The so-called DNA methylation refers to the covalent bond of cytosine at the 5 carbon position of a CpG dinucleotide in the genome combined with a methyl group under the action of DNA methyltransferase. A large number of studies have shown that DNA methylation can cause changes in chromatin structure, DNA conformation, DNA stability, and the way of interaction between DNA and protein, thus controlling gene expression [4].

Dachshund family transcription factor 1 (DACH1) is a newly discovered oncogene located on human chromosome 11 and located at NC-000013.11. It can play an oncogenic role by blocking DNA synthesis in tumor epithelial cells and inhibiting the formation and growth of tumor colonies in the tumor stroma, and is commonly expressed in a variety of normal tissues, with roles in regulating cell proliferation, division, migration, adhesion, and growth, but is silently expressed in a variety of It is commonly expressed in many normal tissues and has a role in regulating cell proliferation, division, migration, adhesion, and growth, but is silently expressed or absent in many malignant tissues [5]. It has been shown that esophageal cancer may be a malignancy with a high frequency of methylation in the promoter region of oncogenes [6]. Therefore, oncogene methylation detection is expected to play a great role in the early screening, disease diagnosis, and efficacy monitoring of esophageal cancer, but there are few studies on oncogene methylation in esophageal cancer. In this study, the methylation-specific polymerase chain reaction (MSP) was used to detect the methylation status of DACH1 in esophageal cancer tumor tissues and to investigate its relationship with the sensitivity of radiotherapy in esophageal cancer patients, to provide a theoretical basis for individualized treatment of esophageal cancer patients.

## 2. Data and Methods

### 2.1. Study Subjects

Seventy patients who received radiotherapy after radical esophageal cancer surgery in the radiotherapy department of The Affiliated Huai'an No.1 People's Hospital of Nanjing Medical University from January 2016 to April 2017 were used as study subjects. The inclusion criteria are as follows: (1) all were diagnosed as esophageal squamous carcinoma by postoperative pathological examination; (2) had not received treatment against esophageal squamous carcinoma before admission; (3) received and completed standard radical radiotherapy according to our treatment standard; (4) KPS score ≥80 and expected survival ≥6 months; and (5) patients could complete the follow-up survey. The exclusion criteria are as follows: (1) those with combined malignant diseases in other sites; (2) those with combined systemic infectious diseases or important organ dysfunction; (3) those with contraindications to radiation therapy; and (4) those who refused to participate in this study. Among them, 39 were male and 31 were female; their age ranged from 42 to 83 years, mean 62.58 ± 10.46 years; lesion site: 28 cases in the upper thoracic segment, 25 cases in the middle thoracic segment, and 17 cases in the lower thoracic segment; tumor length: ≤5 cm 41 cases, >5 cm 29 cases; TNM stage: 28 cases in stage I, 17 cases in stage II, 10 cases in stage III, and 15 cases in stage IV; differentiation degree: 35 cases in highly differentiated and 20 cases in moderately differentiated; the degree of differentiation: 35 cases with high differentiation, 20 cases with middle differentiation, and 15 cases with low differentiation; 24 cases with lymph node metastasis and 46 cases without metastasis. Another 30 normal esophageal mucosal tissue specimens were collected for control. The study was approved by The Affiliated Huai'an No.1 People's Hospital of Nanjing Medical University Ethics Committee, and the patients and their families signed the informed consent form.

### 2.2. Treatment

All patients were treated with radical radiotherapy protocols. Patients were treated with 3D conformal radiotherapy or intensity-modulated radiotherapy under 6 MV X-ray with radiotherapy target areas: gross tumor volume (GTV) and positive lymph nodes (GTVnd), clinical target volume (CTV) including GTV, and The clinical target volume (CTV) includes the GTV and GTVnd, with the upper and lower GTV expanding 2-3 cm and the upper and lower GTVnd expanding 1.0–1.5 cm, both of which are placed 0.8–1.0 cm anteriorly and posteriorly; the planning target volume (PTV) is placed 0.5–1.0 cm anteriorly, posteriorly, and posteriorly based on the CTV. The maximum dose to the spinal cord was ≤45 Gy, the average dose to the heart was ≤30 Gy, and the average dose to both lungs was ≤13 Gy.

### 2.3. Methylation Detection of DACH1

#### 2.3.1. Specimens Were Collected from

All tissues were stored in liquid nitrogen immediately after acquisition and then transferred to a −80°C refrigerator for storage.

#### 2.3.2. Tissue DNA Extraction

Take 30 mg each of cryopreserved cancer tissue, paracancer tissue, and normal esophageal mucosal tissue. Grind well and place in an EP tube. Add 1 ml of DNA digestion solution, shake well, and add 10 mg/ml of proteinase K 50 *μ*l overnight. Add an equal volume of saturated phenol/chloroform (1 : 1) for extraction. Mix well and leave it at room temperature for 10 minutes, then centrifuge at 10 000 rpm. Centrifuge for 10 min, separate the supernatant into a new EP tube (containing 1/10 volume of ammonium acetate and 3 times the volume of −20°C anhydrous ethanol), mix upside down, and centrifuge at 3000 rpm for 10 min. Collect the flocculent precipitate, add 1 ml of 70% ethanol precooled at 20°C, centrifuge at 13 000 rpm for 15 minutes, discard the supernatant, dry the precipitate, add 100 *μ*L DNA rehydration solution, incubate overnight at 4°C, and store in a −80°C refrigerator.

#### 2.3.3. DNA Modification by Sodium Bisulfite

(1) Sulfuration modification of DNA: Take 7 *μ*g of DNA stock solution in an EP tube, add sterilized distilled water to fix the volume to 50 *μ*l, add 5.5 *μ*l of newly prepared NaOH solution (2 mol/L), mix well, and incubate in a constant temperature metal bath at 37°C for 20 minutes, then add 300 *μ*l of DNA treatment solution in turn (10 mmol/L). (2) DNA purification recovery after modification: aspirate the liquid under mineral oil, add 1 ml of DNA purification solution, desalinate according to the procedure of the DNA purification kit, add 3 ml of freshly configured NaOH solution (3 mol/L), and leave it at room temperature for 5 minutes. Add 1 *μ*l of glycogen (10 mg/ml), 17 *μ*l of ammonium acetate (7.5 mol/L), and 3 times the volume of precooled anhydrous ethanol, then place in a refrigerator at −80°C for 30 minutes, centrifuge at 12,000 rpm for 5 minutes, discard the supernatant, add 200 *μ*l of 70% anhydrous ethanol, discard the supernatant, collect the precipitate, and then dry at room temperature. Add 20 *μ*l of sterilized distilled water and store the purified DNA solution overnight at −20°C in a refrigerator at 4°C.

#### 2.3.4. Methylation Assay

A portion of the DNA modified with sodium bisulfite was added to the methylated and unmethylated upstream and downstream primers of DACH1 for PCR amplification. Methylation-specific polymerase chain reaction (MSP) amplification system: 2 *μ*l DNA template, 0.5 *μ*l each of methylation and nonmethylation upstream and downstream primers (200 nmol/L), 11 *μ*l mix, 5 *μ*l ddH_2_ O, and a total of 20 *μ*l. MSP Cycling conditions: predenaturation at 95°C for 5 minutes, denaturation at 95°C for 30 s, annealing at 60°C for 30 s, extension at 72°C for 40 s, a total of 38 cycles, and final extension at 72°C for 10 minutes. Normal human peripheral blood cell DNA treated and untreated with CpG methyltransferase SSSI were used as positive and negative controls, respectively, and the reaction system with sterile deionized water replacing the DNA template was used as PCR. The products were stained with 2.0% agarose gel electrophoresis and ethidium bromide, and the results were observed under a gel imager and photographed. Amplification is negative and the nonmethylated primer amplification of the same sample is positive; the gene is judged not to be methylated [7]. DACH1 methylation positivity rate (%) = number of positive methylation cases/total cases × 100%. The MSP primers were synthesized by Biotech Bioengineering (Shanghai) Co., as shown in Table 1.

### 2.4. Determination of Efficacy

Enhanced CT and X-ray barium meal imaging were performed 1 month after the completion of radiotherapy, and the efficacy was evaluated according to the solid tumor evaluation standard RECIST1.11 [8], which was divided into complete response (CR), partial response (PR), stable disease (SD), and progressive disease (PD). CR + PR was considered sensitive to radiotherapy, and SD + PD was considered insensitive to radiotherapy.

### 2.5. Follow-up

A combination of telephone and outpatient follow-up was used, with follow-up visits every 3 months after the end of radiotherapy to understand the survival status of the affected patients. The follow-up deadline was April 2022. Overall survival (OS) was defined as the time from pathological diagnosis to death or the last follow-up visit.

### 2.6. Statistical Methods

SPSS 22.0 software was used for statistical analysis. Count data were expressed as frequencies and percentages [*n* (%)] using the *χ*^2^ test. The Kaplan–Meier and log-rank tests were used for one-way survival analysis, and multifactor Cox regression models were used to explore the independent influences on radiotherapy sensitivity in patients with esophageal cancer. The test level was *α* = 0.05.

## 3. Results

### 3.1. Comparison of DACH1 Methylation in Each Tissue

The methylation rate of DACH1 in esophageal cancer tissues was higher than that in paraneoplastic and normal tissues, and the difference was statistically significant (*P* < 0.05). The difference was not statistically significant (*P* > 0.05) when comparing the methylation rate of DACH1 in paraneoplastic and normal tissues, as shown in Table 2.

### 3.2. Comparison of DACH1 Methylation between Radiotherapy-Sensitive and Radiotherapy-Insensitive Groups

70 patients with esophageal cancer completed radiotherapy, including 46 radiotherapy-sensitive patients and 24 radiotherapy-insensitive patients. The rate of DACH1 methylation in the radiotherapy-sensitive group was lower than that in the radiotherapy-insensitive group, and the difference was statistically significant (*P* < 0.05), as shown in Table 3.

### 3.3. Relationship between the Methylation Status of DACH1 and Clinicopathological Characteristics of Esophageal Cancer Patients

The methylation rate of DACH1 was higher in esophageal cancer patients with TNM stage (stage III-IV), tumor differentiation degree (hypofractionation), and lymph node metastasis, and the difference was statistically significant (*P* < 0.05). The methylation rate of DACH1 in esophageal cancer patients with different gender, age, lesion site, and tumor length. The differences were not statistically significant (*P* > 0.05), as shown in Table 4.

### 3.4. Analysis of the Relationship between DACH1 Methylation and Radiotherapy Sensitivity and Survival of Esophageal Cancer Patients

The Kaplan-Meier curve showed that the median survival time of patients with DACH1 methylation before radiotherapy was 23 months, which was shorter than the median survival time of patients with DACH1 unmethylation before radiotherapy (36 months), and the difference was statistically significant when comparing the survival curves of the two groups (*χ*^2^ = 7.425, *P* < 0.05), as shown in Figure 1(a). The median survival time of patients in the radiotherapy-sensitive group was 39 months, which was longer than the median survival time of patients in the radiotherapy-insensitive group (25 months), and the difference in survival curves between the two groups was statistically significant (*χ*^2^ = 7.011, *P* < 0.05), as shown in Figure 1(b).

### 3.5. Multifactor Cox Analysis of Radiotherapy Sensitivity in Esophageal Cancer Patients

The results of the multifactor Cox regression model showed that TNM stage (stage III-IV) (HR = 1.961, 95% CI: 1.125 to 2.768), tumor hypofractionation (HR = 1.453, *95%* CI: 1.034 to 2.857), presence of lymph node metastasis (HR = 1.499, *95*% CI: 1.025 to 2.851), and DACH1 methylation (HR = 1.718, 95% CI: 1.067 to 2.596) may increase the risk of insensitivity to radiotherapy in patients with esophageal cancer (*P* < 0.05), as shown in Table 5.

## 4. Discussion

In recent years, the incidence and mortality rates of esophageal cancer have been significantly reduced with the upgrading of treatments, but the overall survival rate is still unsatisfactory. Modern oncology theory suggests that the development of esophageal cancer is a complex process with multifactorial effects, multigene involvement, and multistage development, which is equally closely related to DNA nucleotide sequence alterations (genetics) and epigenetic alterations in addition to environmental factors [9]. Normal DNA methylation is the most studied epigenetic modification mode, and it can maintain gene imprinting, genomic structural stability, *X* chromosome inactivation in females, embryonic development, cell differentiation, and many other functions, whereas abnormal DNA methylation, including overall genomic hypomethylation and hypermethylation of promoter regions, causes disease [10, 11].

The coding genes containing CpG islands are up to 60% in the usual state and are mostly nonmethylated, while CpG island hypermethylation in the promoter region of oncogenes has become a key marker in the carcinogenesis of some tumors and a common mechanism for transcriptional deletion of oncogenes [12, 13]. Studies have shown that the methylation of CpG islands in the promoter region of oncogenes is progressively altered during the carcinogenesis of esophageal squamous carcinoma, and the inactivation of methylation-related genes will have a greater impact on various cell signaling pathways such as DNA damage repair system, apoptosis, and cell adhesion, thus participating in the development of esophageal carcinoma [14]. In this study, the methylation rate of DACH1 in esophageal cancer tissues was higher than that in paraneoplastic and normal tissues, suggesting that methylation of DACH1 exists in esophageal cancer tissues and that this alteration leads to the inactivation of DACH1, resulting in the development of esophageal cancer. DACH1, as an important oncogene, can play an important role in the expression of abnormal transforming growth factor-*β*, Wnt, apoptosis, and other signaling pathways. Its DS structural domain can interact with multiple transcription factors to form transcriptional regulatory complexes and inhibit the expression of the TGF-B signaling pathway, thus suppressing the proliferation of tumor cells [15]. It was found that DACH1 expression was generally reduced in esophageal cancer tissues, and this alteration was due to the regulation of methylation in the promoter region of the gene, while DACH1 expression was upregulated after treating some esophageal cancer cell lines with methylation enzyme inhibitors in vitro [16]. Based on the above analysis, it is easy to find that the hypermethylation status of DACH1 is closely related to the disease progression of esophageal cancer.

Approximately 50% to 60% of esophageal cancer patients receive radiation therapy. However, in clinical work, investigators have noted that patients with esophageal cancer treated with the same radiation therapy did not achieve consistent near term outcomes and prognosis, with significant differences in radiosensitivity, and such interindividual differences in response to radiation therapy may be associated with epigenetic alterations [17]. The results of this study showed that the rate of DACH1 methylation was lower in the radiotherapy-sensitive group than in the radiotherapy-insensitive group, and this result suggested that the sensitivity of esophageal cancer radiotherapy may be related to the methylation status of DACH1. Our analysis suggests that radiation may stimulate esophageal cancer cells to promote high expression of DACH1, which in turn inhibits tumor cell differentiation and achieves a radiotherapy effect, while DACH1 methylation can inhibit DACH1 expression and the inhibitory effect on tumor differentiation is diminished, thus showing radiotherapy insensitivity [18]. In addition, this study analyzed the relationship between the methylation status of DACH1 and the clinicopathological characteristics of esophageal cancer patients and found that the methylation of DACH1 was higher in esophageal cancer patients with TNM stage (stage III-IV), tumor cytodifferentiation, and lymph node metastasis, and this result was consistent with the results of Liu et al. [19], indicating that DACH1 methylation predicted the invasion, This result is consistent with the results of Liu et al., indicating that the methylation of DACH1 predicts the enhanced invasion, differentiation, and metastasis of esophageal cancer tumor tissues and the late TNM stage, while such patients usually have lower radiotherapy sensitivity and poorer recent efficacy. The results of the Kaplan–Meier curve in this study showed that the survival of patients with DACH1 methylation was shorter, and the survival of patients with insensitivity to radiotherapy was also shorter, which indicated that DACH1 methylation and insensitivity to radiotherapy predicted a poor prognosis for esophageal cancer patients. Further multifactorial Cox analysis revealed that TNM stage (stage III-IV), tumor hypofractionation, presence of lymph node metastasis, and DACH1 methylation may all increase the risk of radiation therapy insensitivity and poor prognosis in esophageal cancer patients, suggesting that the methylation status of DACH1 may be used as a predictor of chemotherapy sensitivity and prognosis in esophageal cancer, which may be related to the inhibition of transforming DACH1 by methylation This may be related to the fact that the methylated DACH1 inhibits the transmission of the transforming growth factor-*β* signaling pathway, resulting in the downregulation of the expression of downstream signaling target molecules, which in turn fails to regulate the expression of factors that promote cell division and proliferation [20]. However, the exact mechanism of the effect needs to be confirmed by further in-depth studies and verified in clinical practice [21].

## 5. Conclusion

In conclusion, DACH1 methylation in esophageal cancer may be involved in disease onset and progression, and patients with DACH1 methylation have low sensitivity to radiotherapy and poor prognosis, which is expected to be a new indicator for diagnosis, disease and prognosis assessment, and efficacy monitoring of esophageal cancer.

## Figures and Tables

**Figure 1:** Relationship between the methylation status of DACH1 and radiotherapy sensitivity before radiotherapy and survival of patients with esophageal cancer. (a). Relationship between the methylation status of DACH1 and survival of patients with esophageal cancer before radiotherapy. (b). Relationship between radiotherapy sensitivity and survival of patients with esophageal cancer.

**Table 1:** MSP primer sequences.

Primer name	Primer sequences	Primer length
Methylation primer (M)	5′-GGAAAAAATTATTAGTTTTCGCGGAC-3′	183
	5′-AAACCGAAAACACAAAAATAACGATCG-3′	

Nonmethylated primers (U)	5′-TTTGGAAAAAATTATTAGTTTTTGTGGAT-3′	213
	5′-AAAAAACCAAAAACACAAAAATAACAATCA-3′	

**Table 2:** Comparison of DACH1 methylation in each tissue (*n*, %).

Group	Number of cases	Methylation	Unmethylation
Cancerous tissue	70	22 (31.43)^ab^	48 (68.57)^ab^
Paracancerous tissue	70	2 (2.86)	68 (97.14)
Normal tissue	30	0 (0)	30 (100.00)
*χ* ^2^ value		29.553	
*P*-value		<0.001	

Note. Compared with normal tissues, ^a^*P* < 0.05; compared with paraneoplastic tissues, ^b^*P* < 0.05.

**Table 3:** Comparison of DACH1 methylation between radiotherapy-sensitive and radiotherapy-insensitive groups of esophageal cancer patients (*n*, %).

Group	Number of cases	Methylation	Unmethylation
Radiotherapy sensitive group	46	7 (15.22)	39 (84.78)
Radiation therapy insensitive group	24	15 (62.50)	9 (37.50)
*χ* ^2^ value		16.361	
*P* value		<0.001	

**Table 4:** Relationship between methylation status of DACH1 and clinicopathological characteristics of patients with esophageal cancer (*n*, %).

Clinicopathological features	Number of cases	DACH1		*χ* ^2^ value	*P* value
		Methylation	Unmethylation		
Gender					
Male	39	13 (33.33)	26 (66.67)	0.148	0.700
Female	31	9 (29.03)	22 (70.97)		

Age (years)					
<60	26	7 (26.92)	19 (73.08)	0.390	0.533
≥60	44	15 (34.09)	29 (65.91)		

Lesion site					
Upper thoracic segment	28	10 (35.71)	18 (64.29)	0.735	0.693
Mid-thorax	25	8 (32.00)	17 (68.00)		
Lower thoracic segment	17	4 (23.53)	13 (76.47)		

Tumor length (cm)					
≤5	41	15 (36.59)	26 (63.41)	1.221	0.269
>5	29	7 (24.14)	22 (75.86)		

TNM staging					
Phase I-II	45	7 (15.56)	38 (84.44)	14.731	<0.001
Phase III-IV	25	15 (60.00)	10 (40.00)		

Degree of tumor differentiation					
High differentiation	35	5 (14.29)	30 (85.71)	11.136	0.004
Middle divergence	20	8 (40.00)	12 (60.00)		
Low differentiation	15	9 (60.00)	6 (40.00)		

Lymph node metastasis					
Yes	24	12 (50.00)	12 (50.00)	5.845	0.016
No	46	10 (21.74)	36 (78.26)		

**Table 5:** Multifactor Cox analysis of radiotherapy sensitivity in patients with esophageal cancer.

Factors	*Beta* value	*SE* value	*Wald* value	*HR* value	95% *CI*	*P* value
Gender (male/female)	0.315	0.238	3.867	0.592	0.139∼1.257	0.268
Age (<60 years old/≥60 years old)	0.475	0.274	4.021	0.652	0.147∼1.189	0.317
Lesion site (upper thorax/mid-thorax/lower thorax)	0.562	0.281	4.114	0.821	0.369∼1.408	0.334
Tumor length (≤5 cm/>5 cm)	0.524	0.329	3.048	0.759	0.318∼1.446	0.289
TNM stage (stage I-II/III-IV)	0.671	0.223	15.528	1.961	1.125–2.768	0.006
Degree of tumor differentiation (high/medium/low)	0.702	0.154	14.529	1.453	1.034∼2.857	0.021
Lymph node metastasis (yes/no)	0.821	0.213	16.428	1.529	1.025–2.851	<0.001
DACH1 (methylated/unmethylated)	0.415	0.189	18.271	1.718	1.067–2.596	<0.001

## Data Availability

The simulation experiment data used to support the findings of this study are available from the corresponding author upon request.
